The article "Application of CNN-Based Machine Learning in the Study of Motor Fault Diagnosis" was retracted in 2023. Reasons: results that could not be reproduced; signs of a paper mill; unreliable results or conclusions; concerns about the data.

# Application of CNN-Based Machine Learning in the Study of Motor Fault Diagnosis

**DOI:** 10.1155/2022/9635251

**Published:** 2022-09-05

**Authors:** Xiuyan Peng, Lunpan Wei, Wei Gao

**Affiliations:** College of Intelligent Systems Science and Engineering, Harbin Engineering University, Harbin, Heilongjiang 150001, China

## Abstract

With the development of science and technology, the rapid development of social economy, the motor as a new type of transmission equipment, in the production and life of people occupies a pivotal position. Under the rapid development of computer and electronic technology, manufacturing equipment is becoming larger, faster, more continuous, and more automated. This has resulted in complex, expensive, accident-damaging, and high-impact equipment for electric motors; even routine maintenance requires significant equipment maintenance and maintenance costs. If a fault occurs, it will cause serious damage to the entire equipment and can even have a major impact on the entire production process, leading to a serious economic and social life. In this paper, a CNN-based machine learning fault diagnosis method is proposed to address the problem of high incidence of motor faults and difficulty in identifying fault types. A fault reproduction test is constructed by machine learning techniques to extract vibration time domain data for normal operating conditions, rotor eccentricity, stator short circuit, and bearing inner ring fault; divide the data segment into 15 speed segments, extract 13 typical time domain features for each speed segment; and perform mathematical statistics for fault diagnosis. Compared with the traditional algorithm, the method has more comprehensive feature information extraction, higher diagnostic accuracy, and faster diagnostic speed, with a fault diagnosis accuracy of 98.7%.

## 1. Introduction

As a kind of mechanical equipment to realize energy conversion, electric motor is commonly used in practical production with its simple structure and high operating efficiency, and it has become the most widely used power equipment at present. Due to the specificity of the working principle of electric motor, it is often complicated in structure and harsh in working condition. Usually, its structure is complex and the working conditions are uncontrollable, so the failure rate is high. However, once the failure occurs [1], the normal production and economic efficiency will bring serious impact, and even to the safety of the operator brings a direct threat. Therefore, the implementation of effective fault diagnosis of the motor is essential for its normal operation.

At present, most enterprises still adopt the method of scheduled maintenance for large motors, and the time point of maintenance depends on the accumulated running time of the motor. When the abnormality occurs, the maintenance and repair will be carried out, and this method relies excessively on the experience of engineers [2]. Using any of the abovementioned methods for motor maintenance can no longer meet the current requirements, and the phenomenon of motor overhaul and disrepair still exists widely. Therefore, condition monitoring should be carried out to effectively improve the accuracy of fault diagnosis and condition prediction [3]. The promotion of condition maintenance has become a realistic requirement for enterprise production and an inevitable development trend for equipment management and maintenance work.

The article "Application of CNN-Based Machine Learning in the Study of Motor Fault Diagnosis" was retracted in 2023. Reasons: results that could not be reproduced; signs of a paper mill; unreliable results or conclusions; concerns about the data.

According to the report of EPRI, 53% of the motor failures originate from mechanical causes, such as bearing failure, unbalance, and looseness; 47% from electrical causes, of which 10% originate from the rotor, such as casting defects resulting in unbalanced breath, and broken strips; 37% from the stator winding (see Figure 1, external factors causing the failure include overload, humidity, poor lubrication, and chemical pollution (see Figure 2.

The source of motor failure is mainly divided into four parts, including rotor fault, which accounts for 10%; stator fault, which accounts for 37%; bearing failure, which accounts for 41%; centering problem, which accounts for 12%.

In this paper, by constructing a fault reproduction test, the vibration time domain data of normal operating conditions, rotor eccentricity, stator short circuit, and bearing inner ring fault are extracted, and the data segment is divided into 15 speed cycles, each segment contains 13 typical time domain feature extraction and mathematical statistics for troubleshooting.

## 2. Related Work

### 2.1. Motor Research Review

A large number of studies have been conducted by domestic and foreign researchers on electric motors. The algorithm of RBF kernel function is chosen to diagnose the motor by characterization and parameter optimization in [4]. A parameter estimation algorithm is used to obtain four characteristic parameters of motor faults through the study in [5]. A method to achieve effective fault diagnosis in [6], for the problem that it is difficult to effectively measure and process the fault signal through the research equipment, the method of using wavelet changes to extract the fault feature signal is proposed, which can effectively characterize the real-time health status of the equipment and effectively realize the online health monitoring of the processing equipment.

According to the optimization process of maintenance strategy, motor fault repair can be divided into three types: ex post maintenance, preventive maintenance, and predictive maintenance [7]. Ex post facto maintenance means overhauling after a failure occurs. This strategy has the advantage of saving investment in condition monitoring and avoiding excessive maintenance and is generally used for a small range of noncore equipment [8]. The method has the disadvantage of not being able to predict accidental downtime, which raises maintenance costs in actual production, and the secondary damage to the equipment brings disastrous consequences to the enterprise, resulting in endless equipment disassembly and maintenance, which eventually leads to production losses and management loss [9–11]. Preventive maintenance is, according to a certain time for the interval, called regular maintenance. The strategy has good controllability, and the maintenance time is determined according to the need. In addition, it prevents accident surprises and reduces the possibility of catastrophic accidents, so the number of spare parts can be controlled, thus reducing cost capital [12]. However, failure-free equipment is also frequently overhauled, and the phenomenon of overmaintenance cannot be avoided, bringing sometimes even less benefit than the cumulative damage caused by maintenance, and the strategy does not completely eliminate unplanned downtime, and there is no targeted life analysis and optimization between different equipment. Predictive maintenance means that maintenance is based on equipment condition monitoring [13]. This strategy reduces unplanned equipment downtime by purchasing and using only the spare parts needed for the equipment when needed and repairing only when appropriate, thus achieving no failures without maintenance [14]. However, this method places high demands on monitoring instruments and system construction, and the high costs incurred for monitoring services as well as personnel inputs do not extend the life of the equipment.

The article "Application of CNN-Based Machine Learning in the Study of Motor Fault Diagnosis" was retracted in 2023. Reasons: results that could not be reproduced; signs of a paper mill; unreliable results or conclusions; concerns about the data.

About motor fault diagnosis principle and technology, mainly including, diagnosis principle: motor fault is generally based on vibration, temperature, noise, and other change conditions for diagnosis [15]. In the early stage of motor failure, engineers use sensors to conduct temperature tests on motor take points to initially confirm the type of fault generation, then determine the location of fault generation through noise, and analyze electrical signals through vibration testers to collect data from the motor to determine the location and cause of the fault. This diagnostic method is suitable for minor faults arising from the use of the motor, such as bearing, gear damage, loose structure, alignment problems, poor lubrication and other mechanical aspects of the problem [16]. For complex and serious motor failures, a spectrum analysis instrument can be used to regularly collect data from the load motor and perform time-domain frequency-domain analysis based on current variations and the waveforms obtained. This method can analyze the deterioration trend of motor faults over time through the changing waveforms and current and other parameters [17]. The motor can be disassembled and examined using a high-voltage insulation tester, ohmmeter, and insulation resistance meter to determine the cause of the motor failure. In addition to the above methods, staff can apply the appropriate electrical inspection equipment to test and analyze the insulation structure of the motor, the life of the motor insulation structure, and motor performance factors, so as to further diagnose the motor failure [18]. The electrical circuit and the magnetic circuit form the main part of the motor, and the two work together to transform energy. Motor failure has both electrical causes and mechanical elements; therefore, factory quality, production process, incoming inspection, winding deterioration, bearing lubrication and alignment, unstable grid voltage, excessive load, and other conditions cannot make the motor in good running condition; thus, fatigue accumulation causes damage to the motor [19]. In production life, equipment personnel can choose the corresponding diagnostic methods for fault analysis and elimination based on the basic principles of motor failure.

Based on the above research, the authors of this paper propose to use the fusion of wavelet change and machine learning to carry out fault diagnosis research on electric motors. Through the design of fault reproduction experiments, several typical fault states of motors are restored, and their corresponding vibration signals are measured, and the purpose of diagnosing different states of motors is achieved through signal measurement and processing, combined with the high accuracy of machine learning methods in fault classification.

### 2.2. Introduction to CNN

In the 1960s, Hubel et al. introduced the concept of receptive fields through their studies of cat visual cortex cells, and in the 1980s, Fukushima proposed the concept of a neurocognitive machine based on the concept of receptive fields, which can be seen as the first implementation of a convolutional neural network; a neurocognitive machine that decomposes a visual pattern into many subpatterns (features) and then enters a hierarchical recursively connected feature planes that are processed, and it attempts to model the visual system, so that it can accomplish recognition even when objects are displaced or slightly deformed.

The article "Application of CNN-Based Machine Learning in the Study of Motor Fault Diagnosis" was retracted in 2023. Reasons: results that could not be reproduced; signs of a paper mill; unreliable results or conclusions; concerns about the data.

Convolutional neural network (CNN) is a variant of the multilayer perceptron (MLP). It was developed by biologists Huber and Wiesel in their early work on the visual cortex of the cat. A complex architecture exists for the cells of the visual cortex. These cells are sensitive to subregions of visual input space, which we call receptive fields, in such a way that they cover the entire visual field area in a flat manner. These cells can be divided into two basic types: simple cells and complex cells. Simple cells respond maximally to the pattern of edge stimuli from within the receptive field. Complex cells have a much larger receptive field, which is locally invariant to stimuli from an exact location.

In general, neurocognitive machines contain two types of neurons, namely, sampling elements, which are responsible for feature extraction, and convolutional elements, which are resistant to deformation, involving two important parameters, namely the receptive field, which determines the number of input connections, and the threshold parameter, which controls the degree of response to feature subpatterns. Convolutional neural networks can be seen as a generalised form of neurocognitive machines, which are a special case of convolutional neural networks.

In this application, its CNN training steps are as follows:

Step 1: Upload dataset
Step 2: Input layer
Step 3: Convolutional layer
Step 4: Aggregation layer
Step 5: Convolutional and pooling layers
Step 6: Dense layer
Step 7: Logit layer

### 2.3. Fault Characteristics of Motors

Vibration is a common mechanical fault. Motors, like other mechanical devices, produce a certain amount of vibration when they are in operation. For various models and specifications of electric motors, their vibrations have certain representative and permissible limits. In the event of a motor fault, the amplitude, vibration type, and frequency spectrum will change to a certain extent. Different faults vibrate at different frequencies, so that the working conditions of the motor can be objectively reflected. Through the analysis of the vibration signal, the working condition of the motor can be better understood, thus laying the foundation for the fault diagnosis of the motor. The vibration of an electric motor is caused by a variety of factors, and its occurrence location and characteristics are not the same. The various vibration characteristics of electric motors and the related influencing factors are analysed from both mechanical and electromagnetic aspects.

1. Mechanical vibration: in the case of unbalanced rotor, abnormal rolling bearing, abnormal sliding bearing, and improper installation and commissioning, it can lead to mechanical vibration. Uneven distribution of the weight of the motor rotor can cause a shift in the center position, and the rotation will produce centrifugal force on one side, resulting in different support forces, thus making the motor not work properly. When the rotor is out of balance, its vibration frequency is equal to the rotor frequency and the amplitude increases as the rotor increases. The unbalance of the rotor is caused by the loss or displacement of rotor parts, displacement of rotor coils due to insulation shrinkage, loosening, unbalanced couplings, and the generation of dirt on the surface of the fan and rotor.
2. Electromagnetic vibration: the motor uses the mutual coupling of magnetic fields in the air gap for the exchange of energy, that is, the use of magnetic fields to achieve the transformation of electromechanical energy. When the motor is in operation, the rotor rotates around the inner cavity of the stator and the magnetic field between the stator and rotor interacts to form a rotational force that acts on the stator seat, causing its periodic deformation and vibration. In the case of abnormal stator, abnormal rotor conductor, and uneven gap, the magnetic field of the motor will change, which will cause the vibration characteristics of the frame to change. When the stator is abnormal, its electromagnetic vibration is mainly twice the frequency of the power supply and disappears immediately after power failure.

The article "Application of CNN-Based Machine Learning in the Study of Motor Fault Diagnosis" was retracted in 2023. Reasons: results that could not be reproduced; signs of a paper mill; unreliable results or conclusions; concerns about the data.

## 3. Motor Fault Diagnosis Method

A fault diagnosis method using wavelet variation and machine learning is proposed for the problem such as difficult and complex feature extraction and difficult fault identification. And the bench experiment is carried out to extract the vibration time domain data of normal working condition, rotor eccentricity, stator short circuit, and bearing inner ring fault; calculate the variance contribution rate; and classify the faults by machine learning method with the obtained two-dimensional features.

### 3.1. Motor Fault Feature Extraction

Mechanical vibration exists during motor operation, so the motor with faults is selected for fault reproduction vibration signal measurement. In practice, motor faults are divided into 3 main categories: unbalanced rotor, bent rotor, and loose base, so experiments of motor faults and normal 4 motor states need to be constructed. In the actual operation of the motor, the sources of vibration are more numerous. And any mechanical equipment has inherent mechanical vibration, so it is difficult to effectively extract its corresponding fault feature signal.

The article "Application of CNN-Based Machine Learning in the Study of Motor Fault Diagnosis" was retracted in 2023. Reasons: results that could not be reproduced; signs of a paper mill; unreliable results or conclusions; concerns about the data.

### 3.2. Motor Simulation Test with Different Fault States

A three-phase motor of model HJNl 100L1-4 from Marathon was selected. Different fault reproduction tests were conducted on a university motor test bench. The signals of the four states of the motor were collected using an INV data acquisition system with a sampling frequency of *f*(*s*)=50*Hz* and an acquisition time of *t* = 10 *s*, respectively.

The relevant devices and their performance parameters are as follows: motor HJNl 100L1.4, standard voltage 380 v, standard power 2.2 kw, motor speed l425 r/min, mass 35 kg; acceleration sensor CA-YD-186, frequency range 0.1–6 kHz; signal acquisition system INV303/306; signal adaptor YE3832 IEPE, the output amplitude is (2.5 ± 2.2)V.

The fault simulation test is conducted on the motor. The motors of four state categories were selected for the test. Test plan: the motor end cover and stator outside the installation of acceleration sensors, respectively. All use the contact installation method, using magnets to fix the acceleration sensor on its surface. The signals were acquired by replacing the motors in each of the four states on the fault test bench. A total of 160 (4 × 2 × 20) samples were obtained through the INV data system. Thevibration time domaindata for a certain period of time of 1s for normal operating conditions, rotor eccentricity, stator short circuit, and bearing inner ring fault were first randomlyselected as shown in Figures 3–6.

Then, the normal motor and rotor unbalance time domain waveforms for a period of 1000s were randomly selected, as shown in Figure 7 and 8, respectively.

Comparing Figures 7 and 8, it can be seen that the rotor unbalance vibration is stronger than normal motor, but the difference is not big, so it is difficult to discriminate the fault through vibration signal directly. Therefore, the vibration signal needs to be processed, and the authors of this paper choose the wavelet variation method to process and analyze the signal.

### 3.3. Wavelet Variation Parameters Determination

Before using wavelet variation for signal processing, three parameters *m*, *r*, *N* need to be determined first, usually *m*  = 2, *r*=0.1 ~ 0.25*SD*_*x*_, (where *SD*_*x*_ is the standard deviation of the original data *u*(*i*)), and *N* is 100 to 5000.

### 3.4. Wavelet Variation Feature Vector Extraction

Based on the fault reproduction test, 4 × 2 × 20 vibration samples of the motor are collected, and let each vibration signal be *x*(*i*), so there are *x*(1), *x*(2) …, *x*(160) in total 160 points. The sample values measured at 2 measurement points in a state *i* are shown in *T*_*i*_, *x*_*k*,*j*_ where *j* denotes the measurement point and *k* denotes the *k*th sample of measurement point *j*.

(1) $$\begin{array}{c} T_{i}=\left[\begin{array}{cc} x_{11} & x_{12}\\ \vdots & \vdots \\ x_{20,1} & x_{20,2} \end{array}\right]. \end{array}$$

There is a 20 × 2 sample matrix corresponding to the *i*th state. The corresponding matrix can be obtained by determining each wavelet change value based on (1). By dividing each row, 20 eigenvectors can be obtained. The feature vectors represent the wavelet variation values of the vibration signals corresponding to the 2 measurement points in a certain state. Therefore, there are 20 wavelet variation eigenvectors in a certain state of the motor, i.e. *S*_*i*_=[*E*_*i*,1_, *E*_*i*,2_,…,*E*_*i*,20_]^*T*^, and there are 4 states in the motor simulation test. That is, there are 80 wavelet variation eigenvectors.

The article "Application of CNN-Based Machine Learning in the Study of Motor Fault Diagnosis" was retracted in 2023. Reasons: results that could not be reproduced; signs of a paper mill; unreliable results or conclusions; concerns about the data.

### 3.5. Wavelet Packet Noise Reduction Steps for Signals

In this paper, wavelet packet analysis is used in fault diagnosis to reduce noise. The specific procedures are as follows:

1. The wavelet packet method is used to decompose the signal. Wavelets are selected and the desired level of decomposition is determined, which is then decomposed into wavelet packets.
2. For a given entropy criterion, determine the optimal tree (this step is not essential and can be used selectively for different purposes).
3. Threshold quantization of the decomposition coefficients of the wavelet packet and select a suitable threshold value for it.
4. Perform wavelet packet reconstruction using the low-level decomposition coefficients of the wavelet packet and the quantized coefficients.

## 4. Case Study

Considering that the divided feature vector belongs to a small sample set and the fault type is clear, the SVM algorithm is selected to diagnose the fault.

### 4.1. Support Vector Machine (SVM) Algorithm

The motor fault classification problem is a linear regression problem. Calculated by the following equation:

(2) $$\begin{array}{c} f\left(x\right)=\omega^{T}x+b, \end{array}$$

where *x* is the input vector, *ω* is the weight coefficient, and *b* is the bias.

The fault classification diagnostic function of the support vector machine, which can be expressed in the following equation:

(3) $$\begin{array}{c} \psi \left(\omega ,\xi ,\xi_{i}^{*}\right)=\frac{1}{2}{\left\|\omega \right\|}^{2}+C\sum_{i=1}^{1}\left(\xi_{i}+\xi_{i}^{*}\right), \end{array}$$

where *ω* is the weight coefficient, *C* is the penalty factor, and *ξ*, *ξ*_*i*_^*∗*^ are the upper and lower limits of the slack variables, respectively.

The constraint conditions are given by

(4) $$\begin{array}{c} \text{s}.\text{t}.\left[\left(x_{i}\cdot \omega \right)+b\right]-y_{i}\leq \xi_{i}+\varepsilon ,\\ i=1,2,\ldots ,l, \end{array}$$

where: *ξ*_*i*_ is the relaxation variable, *ω* is the allowable error, *y*_*i*_ is the output corresponding to the *i*th sample [21–25].

The article "Application of CNN-Based Machine Learning in the Study of Motor Fault Diagnosis" was retracted in 2023. Reasons: results that could not be reproduced; signs of a paper mill; unreliable results or conclusions; concerns about the data.

Introducing Lagrange function

(5) $$\begin{array}{c} \sum_{i=1}^{i}\left(\alpha_{i}-\alpha_{i}^{*}\right)=0. \end{array}$$

Using the pairwise principle, Lagrange multiplier method, the pairwise form of the optimization problem can be obtained by substituting (6) into (3) as follows:

(6) $$\begin{array}{c} {\underset{\alpha ,\alpha^{*}}{\max}}^{w}=-\frac{1}{2}\sum_{i=1}\sum_{j=1}\left(\alpha_{i}-\alpha_{i}^{*}\right)\left(\alpha_{j}-\alpha_{j}^{*}\right)K\left(x_{i},x_{j}\right)+\sum \left[\alpha_{i}\left(y_{i}-\varepsilon \right)-\alpha_{i}^{*}\left(y_{i}+\varepsilon \right)\right]. \end{array}$$

That is, the output of the support vector machine is as follows:

(7) $$\begin{array}{c} f\left(x\right)=\sum_{i=1}\left(a_{i},a_{i}^{*}\right)K\left(x_{i},x\right)+b, \end{array}$$

where *a*_*i*_, *a*_*i*_^*∗*^ is the Lagrange multiplier; *b* is the bias.

### 4.2. Fault Diagnosis

The process of building a multifault classifier using support vector mechanism is shown in Figure 9. The model is as follows:

(8) $$\begin{array}{c} f_{F}\left(x\right)=\text{sign}\left[\sum_{n}y_{i}\alpha^{*}K\left(x_{i}\cdot x_{j}\right)+b^{*}\right], \end{array}$$

where *K*(*x*_*i*_, *x*_*j*_) is the kernel function, and the radial basis kernel function is chosen with the expression.

(9) $$\begin{array}{c} K\left(x,y\right)=\text{exp}\left(-\frac{{\left\|x-y\right\|}^{2}}{2\sigma^{2}}\right), \end{array}$$

where *σ* is the parameter that controls the width of the kernel function.

The SVM is used to diagnose 4 types of faults in motors; 20 groups of each of the 4 states, i.e., a total of 80 groups of feature vectors. Then, the test samples are used for validation. For each state, 10 sets of test data are selected and tested four times. The wavelet variation values for each state category of the motor are shown in Table 1.

MATLAB 7.0 was chosen to set up the corresponding SVM program for diagnosis, and the penalty parameters of the model were *C*_*i*_, kernel width *σ*_*i*_ (*i*  = 1, 2, ⋯, 9). The highest training accuracy was achieved using training samples in MATLAB at *C*_*i*_  = 100, *σ*_*i*_  = 1. The data in Table 1 were validated and the classification results show that the SVM classification model was used to diagnose the test samples with an accuracy of 97.5%, and only one rotor bend was misclassified as a loose base fault [26].

### 4.3. Comparison of Different Fault Diagnosis Methods

The commonly used improved BP neural network diagnosis method is selected to train the sample set of wavelet variation feature quantity of the motor. The validation samples are used to verify and compare the diagnosis results with SVM. The commonly used 3-layer BP neural network model is selected to construct the motor fault classification prediction model as shown in Figure 10.

The article "Application of CNN-Based Machine Learning in the Study of Motor Fault Diagnosis" was retracted in 2023. Reasons: results that could not be reproduced; signs of a paper mill; unreliable results or conclusions; concerns about the data.

The validation samples are input into the BP classification model for diagnosis, and the classification results show that a normal motor condition is mistaken for a rotor unbalance fault. A rotor bending fault is mistaken for a loose base fault. A loose base fault was mistaken for a rotor bending fault, and a total of three state categories were misclassified, with an accuracy rate of 92.5%.

The results of diagnostic classification for different types of vibrations for normal operating conditions, rotor eccentricity, stator short circuit, and bearing inner ring faults are shown in Table 2. The mixture matrix output from the table shows that the faults are classified more accurately, and the diagnostic accuracy in this case is as high as 98.97%.

## 5. Conclusion

The motor vibration signal feature extraction is difficult and complex, and fault identification is difficult. The motor experiment platform is used to extract the motor normal and fault conditions data, and a motor fault diagnosis model based on wavelet transform and machine learning is proposed. The method is applied to the diagnosis and maintenance of motor faults. Based on failure analysis, reliability maintenance is performed to avoid overmaintenance and undermaintenance of equipment, early detection of equipment failures, and better control of spare parts.

Wavelet analysis can decompose the signal into wavelet expanded fundamental functions, so that the signal can be locally refined in the high- and low-frequency parts, while maintaining the time-frequency characteristics of the signal, thus making the signal have better time-frequency characteristics, which can effectively identify the signal and thus achieve fault diagnosis of the signal. In this paper, wavelet analysis techniques are used for fault simulation of electric motors. Wavelet analysis is a new diagnostic technique.

There are two methods of combining wavelet analysis and neural networks.

1. Loosely combined: wavelet analysis is a preprocessing method for traditional neural networks, which provides feature vectors for neural networks and trains and diagnoses them. The two are closely but independently related.
2. Closely integrated: feedforward networks based on wavelet analysis. The basic idea is to use wavelet elements to substitute for neurons, i.e., the activation function is the wavelet function base, and the scale and translation parameters of the wavelet function replace the corresponding input layer to the hidden layer weight and hidden layer threshold [20].

The article "Application of CNN-Based Machine Learning in the Study of Motor Fault Diagnosis" was retracted in 2023. Reasons: results that could not be reproduced; signs of a paper mill; unreliable results or conclusions; concerns about the data.

## Figures and Tables

**Figure 1:** Motor failure source.

**Figure 2:** External factors causing failure.

**Figure 3:** Normal working condition.

**Figure 4:** Rotor eccentricity.

**Figure 5:** Stator short circuit.

**Figure 6:** Bearing inner ring failure.

**Figure 7:** Normal motor time domain waveform.

**Figure 8:** Time domain waveform of rotor unbalanced motor.

**Figure 9:** Flow of SVM to build a fault classifier.

**Figure 10:** Improved BP neural network classification model.

**Table 1:** Wavelet variation values for each state category of the motor.

Category	Group 1		Group 2		Group 3		Group 4	
	Measurement point 1	Measurement point 2	Measurement point 1	Measurement point 2	Measurement point 1	Measurement point 2	Measurement point 1	Measurement point 2
1	0.551	0.521	0.698	0.961	0.691	0.887	0.556	0.507
2	0.785	0.597	0.731	0.525	0.778	0.546	0.811	0.621
3	1.078	1.017	0.856	0.965	0.871	0.712	1.126	0.987
4	0.997	0.879	0.856	0.941	0.871	0.756	0.883	0.958

**Table 2:** Mixing matrix of classifier output.

Prediction	Normal	Rotor eccentricity	Stator short circuit	Bearing inner ring
Normal	28	0	0	0
Rotor eccentricity	0	19	0	0
Stator short circuit	1	0	25	0
Bearing inner ring	0	0	0	25

## Data Availability

The dataset used in this study can be obtained from the corresponding author upon request.
